# Effect and Mechanism of Traditional Chinese Medicine Exercise Therapy on Stroke Recovery

**DOI:** 10.1155/2023/5507186

**Published:** 2023-02-21

**Authors:** Cunxiao Guo, Yuanwang Wang, Shuang Wang, Shouyao Zhang, Xiantao Tai

**Affiliations:** School of Acupuncture, Tuina and Rehabilitation, Yunnan University of Chinese Medicine, Kunming, Yunnan 650500, China

## Abstract

Stroke is currently the second largest contributor to disability-adjusted life years (DALYs) in developing countries, and it is the third largest contributor to DALYs in developed countries. It requires a large number of resources from the health care system every year, which places a great burden on society, families, and individuals. The treatment of traditional Chinese medicine exercise therapy (TCMET) during stroke recovery has become a hot topic of current research due to its few adverse events and high efficiency. This article sorts out the latest progress of TCMET on the recovery of stroke through the review method and explores its role and mechanism based on existing clinical and experimental studies. TCMET treatment of stroke recovery mainly includes Tai Chi, Baduanjin, Daoyin, Yi Jin Jing, five-fowl play, and six-character tips, which can effectively improve motor function, balance and coordination ability, cognitive dysfunction, nerve function, depression or emotional state, daily living ability, and so on after stroke. The mechanisms of stroke treated by TCMET are discussed, and deficiencies in the literature are discussed and analyzed. It is hoped that some guiding suggestions will be provided for future clinical treatment and experimental studies.

## 1. Introduction

Stroke disease is also known as stroke. It is a type of disease that is mainly manifested by sudden coma, unconsciousness, half-body failure, tongue tilting, and unfavorable speech [1]. It is equivalent to the cerebrovascular accident (CVA) in modern medicine. According to the pathological results, stroke is divided into ischemic stroke, cerebral hemorrhage, subarachnoid hemorrhage, and mixed stroke. According to the 2020 Chinese Stroke Association Guidelines for Clinical Management of Cerebrovascular Diseases, stroke is clinically divided into three distinct stages: the acute stage, the recovery period, and the sequelae period. The acute phase refers to the onset of illness within 1 month. The recovery period is 1 month to half a year after the onset of the disease, and half a year later is the sequelae period [2].

Stroke is currently the second largest contributor to disability-adjusted life years (DALYs) in developing countries, and it is the third largest contributor to DALYs in developed countries [3]. Globally, 132.1 million DALYs have been lost [4]. This requires significant resources from the healthcare system [5]. The incidence of stroke varies greatly according to the age structure of the population under study. With age, the incidence increases dramatically in both men and women. The risk of disease in children under 15 years of age is 1 in 100,000, while the risk of disease in people aged 85 years and older is 1 in 33. The incidence of stroke from the age of 55 to the age of 84 more than doubles every decade [6]. Stroke deaths in China in recent years have accounted for one-third of the total number of stroke deaths worldwide [7, 8]. There are certainly regional differences in the incidence of the disease, mostly in the northern and central regions. About 70% of stroke survivors have some degree of disability, including physical and mental disabilities, mobility restrictions, and participation restrictions [9]. This increases the burden of stroke-related disabilities in China and other countries around the world, putting enormous pressure on society, families, and individuals. With the advent of an aging population, these problems will become more pronounced in the future. How to solve the problem of disability caused by stroke will become the direction of continuous exploration in this research field.

Traditional Chinese medicine exercise therapy (TCMET) is also known as Gong Fa. Under the guidance of holism in traditional Chinese medicine (TCM) and treatment based on syndrome differentiation, there are certain exercise principles and operating methods, and through the coordination and unification of exercise, breathing, consciousness, and self-tuina, that is, the combination of “body adjustment, heart adjustment, and pranayama,” a kind of exercise therapy is used to prevent and treat diseases and strengthen the body. During the exercise, it is required to relax the body and mind, pay attention to softness and rigidity, and static braking. In the state of relaxation and naturalness, body movement is used to practice shape, and breathing exercise is used to practice qi, while mind guidance is used to restore the normal operation of qi and blood around the body, so that the body can recover. TCMET is an important part of TCM and belongs to a kind of aerobic exercise of active exercise, mainly including Tai Chi, Baduanjin, Daoyin, Yi Jin Jing, five-fowl play, six-character tips, Shaolin kung-fu, Relaxation exercise, and Standing pile exercise. For the study of stroke disease, the ancient Chinese physician Chao Yuanfang quoted many Daoyin methods in the “Health Care Formula Guide Method” in the “General Treatise on Causes and Manifestations of All Diseases” to treat stroke disease. Liu Wansu attaches great importance to the restoration of the motor function of stroke hemiplegia by TCM and early Daoyin tuina. TCMET is convenient, economical, and rarely causes adverse events; the safety, efficacy, and fall rates were also confirmed by literature studies [10–12]. Therefore, TCMET's treatment of stroke disease has attracted more and more attention.

## 2. Search Strategy and Literature Screening

### 2.1. Search Strategy

The literature was searched in PubMed, Web of Science, Embase, Cochrane library, China national knowledge infrastructure (CNKI), ChongqingVIP, and Wanfang database, from the establishment of the library to Aug 29, 2022, through the keywords “Traditional Chinese Medicine Exercise Therapy,” “Tai chi,” “Baduanjin,” “Daoyin,” “Yi Jin Jing,” “five-fowl play,” “six-character tips,” “Shaolin kung-fu,” “Health care exercises,” “Relaxation exercises,” “Standing pile exercises,” and “Stroke” and adjusted according to different databases. The search strategy of the PubMed database is shown in Table 1.

### 2.2. Literature Screening

A total of 2571 articles were identified in the search, and 228 articles were deemed potentially relevant through the exclusion of the title and abstract. There were 71 articles through reading the full text to exclude repeated publications, research proposals, abstracts, case studies, and conference papers. The full text cannot be found and it is still in clinical trials. The literature clearly did not belong to the stroke recovery period. Among them, there are 24 articles on Tai Chi, 18 articles on Baduanjin, 9 articles on Daoyin, 5 articles on Yi Jin Jing, 2 articles on five-fowl play, 10 articles on six-character tips, and 3 articles on relaxation exercises (Figure 1).

## 3. Research Status

Judging from the published literature, the hot spots of research in the past decade have mainly focused on the treatment of the stroke recovery period with TCMET. By choosing this stage of treatment and the introduction of Western medical rehabilitation into China in the 1970s and 1980s and the gradual development of traditional Chinese medicine rehabilitation, the treatment of stroke has placed more and more emphasis on the grasp of the time window. Through clinical studies, the earlier the intervention in traditional Chinese and Western medicine rehabilitation, commonly known as early introduction, the more beneficial it is to the patient's later recovery. Multidisciplinary cross-fusion treatment has become a trend in stroke treatment. TCMET plays a role in the recovery period of stroke with its unique advantages. At present, more research studies are being conducted on Tai Chi, Baduanjin, Daoyin, Yi Jin Jing, five-fowl play, six-character tips, and Relaxation exercises. The summarized current status of TCMET in the recovery period of stroke is shown in Tables 2–7.

From Table 3, Tai Chi uses the simplified 24 forms issued by the General Administration of Sports of China in 2003 and improves on this basis, choosing a single type of exercise such as Tai Chi Yunshou or choosing the 8 postures that are most commonly used for stroke patients. The 8 postures are commencing, step back and whirl arms, knee hugging and twist step, wild horse mane, yunshou, hand waving pipa, picking the tail, ending posture, etc., which include moving forward, backward, left, and right from the fixed step. It also emphasizes the “waist as the axis” to drive the movement training of upper limbs, hips, knees, and ankles. During the practice, the waist and hips are required to be loose and heavy, with breathing exercises..

In the specific practice, attention is paid step by step to specific exercises, from easy to difficult, practiced in stages, and certain protective measures are taken. The intervention time was 20–60 minutes each time, 1-2 times a day and 2–5 times a week. Some literature studies used a combination of group exercises and individual exercises, and the total intervention time was half a month to 6 months. In terms of clinical efficacy, it mainly improved motor function, balance ability, cognitive impairment, neurological function, daily living ability, emotion regulation, cardiopulmonary function, safety, and fall prevention in stroke patients, and it was reported that with the extension of intervention time, the effect was more significant. From the perspective of literature quality, except for one piece of the literature that is unclear whether to use randomized control, the rest of the literature used randomized controlled trials, compared the baseline data of the literature, and recorded the shedding cases, so the results of the included literature studies were recommended.

From Table 4, Baduanjin refers to the “Fitness Qigong Baduanjin” standard issued by the General Administration of Sports of China in 2003 [83], and the Eighteen section brocade is a training method that combines Tai Chi, Baduanjin, and modern fitness exercises. The included literature mainly used Baduanjin or eighteen sections brocade combined with other methods for the treatment of stroke, and the efficacy was significantly better than that of Baduanjin alone or eighteen section brocade. The improvement after stroke is mainly in motor function, balance function, cognitive function, depression after stroke, and daily living ability.

From the perspective of intervention time, compared with Tai Chi, the intervention time of Baduanjin is shorter, generally 20–30 minutes each time, generally once a day in the morning and evening, 40–50 minutes 3 times a week, and the intensity of exercise is in line with the aerobic activity intensity recommended by the American College of Sports Medicine and the American Heart Association for the health of the elderly in 2007 [84]. In terms of the evaluation of literature quality, the included literature all adopted the randomized control method, but there were certain confounding factors due to the combination of multiple methods. The insufficient sample size and a wide range of centers affected the results.

It can be seen from Table 5 that the choice of Daoyin is mainly caused by causes and manifestations of all diseases, which reflect the combination of breath, heart, and body adjustment. Sitting, standing, and horizontal training for different parts can be adopted. The curative effect of Daoyin combined with basic rehabilitation is better than simple basic rehabilitation. The curative effect of stroke is mainly on motor function, balance and coordination ability, daily living ability, and so on. The safety and fall prevention of stroke have not been found in the relevant literature. The total intervention time is relatively short, and the relationship between extended practice time and efficacy remains to be verified.

It is concluded from Table 6 that the six-character tips mainly adopt the fitness qigong six-character tips of the General Administration of Sports of China [85], and some literature combines Daoyin on this basis [86], which can be exercised step by step in supine, sitting, and standing positions. The treatment of stroke is mainly to improve the patient's lung and respiratory function, speech disorders, and so on, and the efficacy of the combination of other methods is significantly better than that of other methods alone. One piece of literature on the source of the case involved a multicentre study [64], but there were limitations and the overall intervention time was short.

From Table 7, it can be concluded that Yi Jin Jing, five-fowl play, and Relaxation exercises are the three TCMETs with the least amount of literature research and the total intervention time is short, which mainly improves motor function and daily living ability of stroke patients. The efficacy of combination with other methods is better than that of other methods alone.

Subgroup analysis of each TCMET therapy is conducted in Tables 3–7. Different TCMETs have common effects on stroke recovery, which also have different characteristics. The summarized efficacy and frequency of TCMET on stroke recovery are shown in Figure 2.

It can be seen from Figure 2 that Taichi and Baduanjin have conducted extensive studies, and TCMET has improved motor function after stroke. Daoyin is mainly used to improve balance and coordination ability and daily living ability in addition to motor function. Besides, Baduanjin has conducted more studies on cognitive function, depression, and emotional state after stroke. Studies on six-character tips are mainly used in lung function and speech disorders. There is relatively little literature on Yi Jin Jing, five-fowl play, and relaxation exercises. Only Taichi and Baduanjin are involved in safety evaluation. However, only Taichi has a special literature study on fall prevention in TCMET.

From the above research and analysis of TCMET on the recovery period of stroke, its efficacy in combination with other therapies is worthy of recognition, which is a useful supplement of modern Western medicine rehabilitation in the recovery period of stroke and is worthy of promotion and application. Subsequent studies were provided in terms of the use, sample size, intervention time, and tendency of each therapy to facilitate function recovery during stroke recovery.

## 4. Mechanism Discussion

### 4.1. To Explore the Mechanism of TCMET from Brain Function Remodeling

#### 4.1.1. From the Functional Structure of the Brain

From the cortex research, Chen Yiyun and Liu believe that stroke patients with hemiplegia actively and consciously practice such as Baduanjin can enhance the activity of the motor center of the human brain cortex and increase the excitability of nerve cells [87]. Liu and Li found that the cerebral cortex was in a special state during the Daoyin exercise, which may be one of the mechanisms of its influence on brain function. In addition, it was also found that skin temperature changes significantly in the process of Daoyin exercise, suggesting that Daoyin exercise can affect autonomic nervous function [88]. Zhu found that specific Daoyin techniques can activate specific areas of the cerebral cortex and promote plastic changes in the central nervous system, and it is believed that the active use of limbs can cause plasticity changes in the function of the brain's motor cortex [89]. From the study of brain gray matter, Ye is based on voxel morphological analysis, and by comparing MRI before and after treatment, it is believed that Baduanjin's effect on gray matter volume in patients with mild cognitive impairment (MCI) is significantly related to the changes in the gray matter structure in the right middle temporal gyrus, the right middle occipital lobe, and the right posterior cerebellar lobe [90]. Based on multimodal magnetic resonance imaging, Lu explored the effect of Tai Chi exercise on cognitive function and believed that Tai Chi tends to adjust the functional connectivity of the brain's default mode network and change the structure of white matter fibers [91]. In a study published in 2012 by Xue et al. in Professor Chen Lidian's team, participants were scanned by resting-state fMRI before and after the 12-week Tai Chi and Baduanjin practice interventions, and the memory function of the subjects was evaluated, aiming to explore whether they could improve memory function and regulate the resting function connection of the hippocampus. The results showed that both Tai Chi and Baduanjin could significantly enhance the memory function of the participants, and the strength of the functional connection between the bilateral hippocampus and the medial prefrontal cortex in the Tai Chi group increased significantly. This change in functional connectivity has a significant correlation with the improvement of memory function in participants, and the intrinsic effect mechanism of Tai Chi in improving memory function is partially illustrated at the level of the central nervous system [92].

#### 4.1.2. Study the Effects of Brain Waves

Chen Chi's research on the effect of fitness qigong six-character tips on brain waves in patients with mild cognitive dysfunction, from the analysis of brain waves (EEG) before and after practice, shows that the approximate entropy is significantly reduced at the beginning of 1 month of practice, the EEG tends to be orderly, and the approximate entropy is still slightly reduced after 3 months of practice, indicating that insisting on practicing fitness qigong six-character tips can keep brain waves more orderly, manifested as memory loss and improvement, improved ability to respond to things, and a calm mood [93].

#### 4.1.3. From Neuromodulation Studies

Zhao et al. found that the “Six-step” Daoyin exercises can stimulate the potential of the central nervous system, and the Daoyin therapy method can clearly improve the motor muscle signal intensity of the quadriceps, and under the guidance of this feedback technology, the patient's exercise program can be gradually re-established. The study also used feedback techniques to show that Daoyin therapy can stimulate people's “thoughts” during the rehabilitation process, thereby promoting the rehabilitation of specified movements to a certain extent [94].

#### 4.1.4. Blood Flow Studies from the Brain

Li et al. observed the circulatory state of brain blood circulation in patients after Daoyin therapy, and the cerebral blood flow chart of patients after Daoyin therapy showed that the blood inflow time was shortened and the tension of blood ducts decreased significantly, indicating that Daoyin therapy can improve the brain blood flow chart, improve blood duct elasticity, and increase cerebral blood volume, particularly vertebrobasilar volume [95].

#### 4.1.5. Study on Changes in Cerebral Blood Oxygen

Qiang et al. measured the brain oxygen metabolism state of a senior Shaolin kung-fu exerciser during exercise by near-infrared spectrophotometry, and the amount of oxygenated hemoglobin was slightly reduced compared with that of the quiet sitting position during the Shaolin kung-fu exercise, and the total hemoglobin amount was almost unchanged. The ratio of oxygenated hemoglobin to oxyhemoglobin in the total hemoglobin volume during the Shaolin kung-fu exercise decreased slightly, and the amount of oxyhemoglobin increased slightly. In terms of oxygen saturation, compared with the quiet sitting position before the Shaolin kung-fu exercise, the Shaolin kung-fu exercise is only reduced by about 1-2%, which cannot be said to have changed significantly. In experiments with senior Shaolin kung-fu exercisers, despite the intensity of isotonic muscle contractions, the total amount of hemoglobin and oxygen saturation in the brain have been maintained within the physiological range. This suggests that the “Natural respiration” method practiced through long-term exercise can promote the very economical oxygen consumption of brain tissue, effectively inhibiting the increase in the amount of deoxyhemoglobin in the blood. Correct, moderate Shaolin kung-fu exercises do not affect the homeostasis of the human environment but can improve the oxygenation capacity of brain tissue [96].

### 4.2. To Explore the Mechanism of TCMET at the Molecular Level

Wang Qian et al. discussed the mechanism of eighteen-section brocade combined acupuncture treatment to improve exercise quality and motor function of patients from the levels of serum matrix metalloproteinases-9 (MMP-9), erythropoietin (EPO), and homocysteine (Hcy). In normal brain tissue, EPO is hardly expressed, but its content is significantly increased in stroke and can be used as a marker of brain damage [97]. HCY is a risk factor for ischemic stroke and atherosclerosis. The study found that MMP-9 is closely related to the structure of the blood vessel wall and the permeability of the blood-brain barrier, which can reflect the edema area and the degree of cerebral infarction in stroke patients. The serum MMP-9, EPO, and Hcy levels in the observation group were significantly lower than those in the control group, indicating that acupuncture combined with eighteen-section brocade could reduce brain injury by reducing serum MMP-9, EPO, and Hcy levels [49]. In addition, some researchers have significantly reduced the urine uric acid content before and after practicing standing pile exercises, which shows that the synthesis of nucleic acids is greater than the decomposition during the exercise, and then the synthesis of nuclear proteins can be introduced to be greater than the decomposition. Whether the resynthesis rate of nuclear protein is accelerated or the decomposition rate of nuclear protein is slowed down during practice, the body will enter a state of energy storage. In turn, it will have a good impact on the function of various organs in the human body. It is believed that the clear-eyed, energetic self-proprioception that occurs after practicing is related to this good effect of influence [98].

### 4.3. To Explore the Mechanism of TCMET from the Changes in Lung Ventilation

Ding et al. explored the mechanism of six-character tips in the treatment of respiratory control ability in patients with motor speech disorder after stroke by comparing six-character tips with traditional breathing training. Its mechanism may be the same as the “six-character tips” which emphasizes the simultaneous training of breathing and pronunciation. Breathing pronunciation is gentle, slow, and uniform, in fact, a low-load, slow-rate breathing training. It is easier to activate the main respiratory muscle group composed of slow muscle fibers than simple respiratory muscle reinforcement training, and it is not easy to cause fatigue and does not cause excessive tension in the vocal cords [64]. In addition, the vocalization method of the “six-character tips” is conducive to the stabilization of subglottic pressure, providing sufficient airflow for vocal cord vibration, ensuring the duration and tone of laryngeal pronunciation, and gradually adjusting the patient's breathing mode to abdominal breathing during training, which helps to enhance the patient's respiratory function and provide continuous and stable respiratory airflow support for pronunciation [99]. Moreover, the “six-character tips” guided action can fully mobilize the respiratory muscles and increase the amplitude of abdominal movement before and after and the range of movement of the diaphragm up and down, which is conducive to increasing the volume of the chest cavity and lung capacity [99, 100]. Some studies have further shown that when training the “Xu” word in the six-character tips of breathing, the air tract and extrathoracic resistance of the body can be increased when exhaling, and the squeeze of the airway by the pressure in the chest can be reduced through this way. The collapse of the small airway and the premature closure of the bronchi are avoided, and the residual air volume in the lungs is reduced, so that the phenomenon of airflow obstruction is reduced, and the role of improving the lung function of the body can be achieved [72]. Some researchers have used Tai Chi to regulate post-stroke cardiopulmonary function by means that the heart rate variability (HRV) of long-term Tai Chi practitioners will be greatly improved. Secondly, the abdominal breathing of Qi Shen Dantian during the long-term practice of Tai Chi not only exercises the respiratory muscles, but also strengthens the depth of breathing, expands the lung capacity, improves the microcirculation system, improves the gas exchange capacity, and has a more obvious effect of increasing the velocity max [22].

In summary, the above studies explore the mechanism of TCMET in stroke treatment from the aspects of brain function remodeling, molecular mechanism, and lung ventilation change mechanism, and prove how TCMET plays a role in stroke treatment. However, the research on the mechanism of action is still relatively weak, and the research on the mechanism needs to be further strengthened if TCMET is to be promoted and applied during the recovery period of stroke.

## 5. Trend of Development

The characteristic of TCM is holism and treatment based on syndrome differentiation. TCMET such as Tai Chi, Baduanjin, Daoyin, Yi Jin Jing, six-character tips, Relaxation exercises, Shaolin kung-fu, and Standing pile exercises mentioned in this article reflect the advantages of TCM through body adjustment, heart adjustment, and pranayama, which can adjust the motor function, balance and coordination ability, and overall disease resistance and rehabilitation ability of stroke patients from multiple levels and angles, which is consistent with the overall rehabilitation and comprehensive rehabilitation goals of stroke rehabilitation and is worthy of further promotion and application. TCMET has achieved some success in the study of the stroke recovery period. However, there are still several issues that merit further in-depth study. For example, in the design of clinical trials, TCMET is difficult to blind, and most studies use evaluator blinding; the sample size of the trial is too small, and further large-sample studies are needed to further confirm the reliability of the data; in terms of inclusion standards, it is difficult for patients with poor motor function and balance function to participate in the trial. The measurement-efficiency relationship of intervention time needs further follow-up and study; there is no completely unified standard for TCMET intervention during stroke recovery. From the analysis of each subgroup in TCMET, most of them used TCMET combined with other drugs, Western medicine rehabilitation, and other methods, and there were many confounding factors and certain limitations. There is relatively insufficient research on safety evaluation and fall prevention; in terms of evaluation standards, most of them are scales, with certain subjectivity; the discussion of mechanism is relatively weak; and further research on the intrinsic characteristics and effect mechanisms of each TCMET, at the molecular level and even deeper levels, needs to be further developed.

In the future, TCMET's prevention and treatment of the stroke recovery period will need to overcome the shortcomings of existing research based on artificial intelligence and big data technology, combined with different TCMET characteristics and the development of different stages of multiexercise or partial stereotype integration of unified standards for TCMET to stroke recovery period research to provide evidence-based medical evidence, multilevel, large sample, multicenter research, and from stroke recovery period to subacute stage transition research, so that more stroke patients can receive timely and early intervention in TCMET treatment. Let this therapy become an effective method for the prevention and treatment of stroke diseases in countries around the world. The burden of stroke is shared by society, families, and individuals.

## Figures and Tables

**Figure 1:** The flow chart of literature screening.

**Figure 2:** The therapeutic effect and the frequency figure of TCMET on recovery of stroke.

**Table 1:** Search strategy for the PubMed database.

Search term	
#1	“Taijiquan”[mesh]
#2	“Tai Chi” OR “Tai Ji” OR “Taiji” OR “Tai Chi Chuan”
#3	#1 OR #2
#4	“Baduanjin” (mesh)
#5	“Daoyin” (mesh)
#6	“Yi Jin Jing” (mesh)
#7	“Five-fowl play” (mesh)
#8	“six-character tips” OR “Liu Zi Jue qigong” (mesh)
#9	“Shaolin kung-fu” OR“Shaolin neigong” (mesh)
#10	“Health care exercises” (mesh)
#11	“Relaxation exercises” (mesh)
#12	“Standing pile exercises” (mesh)
#13	“Traditional Chinese medicine exercise therapy” (mesh)
#14	“Stroke” (mesh)
#15	#3 OR #4 OR #5 OR #6 OR #7 OR #8 OR #9 OR #10 OR #11 OR #12 OR #13
#16	#14 AND #15

**Table 2:** General view of all therapeutic approaches.

Therapeutic approaches/sample number (*n*)	Specifications	Efficacy	Refs
Tai Chi (*n* = 1716)	Based on ancient Chinese philosophical ideas such as the theory of yin and yang and the principle of Tai Chi, it is a traditional boxing technique that integrates functions such as temperament, physical fitness, and technical confrontation	Treating the symptoms and signs during the recovery of stroke	[11, 13–35]
Baduanjin (*n* = 1505)	Baduanjin is a fitness method invented in ancient China. There are eight beautiful and smooth movements such as “Jin,” which is a set of exercises for internal exercises of “Jing, Qi and Spirit” and external exercises for preventing and treating diseases, strengthening the body, and improving physical strength	Treating the symptoms and signs during the recovery of stroke	[36–53]
Daoyin (*n* = 718)	Daoyin is the earliest and most distinctive exercise method in many therapies of TCM, which is a way of organically combining breathing, body movement, idea guidance, and self-tuina, which plays a unique role in health care, disease treatment, and rehabilitation	Treating the symptoms and signs during the recovery of stroke	[54–62]
Six-character tips (*n* = 828)	six-character tips is a set of tuna health care methods handed down in ancient China, focusing on breathing and exhaling using “Xu, He, Hu, Xi, Chui, Xi,” the specific pronunciation of the six characters, mouth training to affect the operation of different organ meridian qi and blood, supplemented by corresponding body movements and ideas, and then achieving the purpose of strengthening the body and maintaining health and rehabilitation	Treating the symptoms and signs during the recovery of stroke	[63–72]
Yi Jin Jing (*n* = 601)	Yi Jin Jing originated from the ancient Chinese health care guidance technique, through the use of subjective energy, a comprehensive exercise of self-body and mind, changing the bones and muscles, making them a strong set of traditional exercises. It uses a certain posture to induce breathing and gradually strengthens the function of the tendons and internal organs	Treating the symptoms and signs during the recovery of stroke	[73–77]
Five-fowl play (*n* = 120)	Five-fowl play is an ancient traditional exercise that imitates the movements of five animals, namely tigers, deer, bears, apes, and birds (cranes), and is a guiding method for health care and strengthening the body	Five-fowl play can significantly improve the motor function, balance function, and ability of daily living in patients with stroke hemiplegia	[78, 79]
Relaxation exercises (*n* = 209)	Relaxation exercises are a kind of meditation exercise, which organically combines the three practice methods of mind, breathing, and posture and adopts postures such as “standing, sitting, and lying down” to relax various parts of the body from the head to the toe, from the top to the bottom, to adjust the whole body to a comfortable, relaxed, and natural state	Treating the symptoms and signs during the recovery of stroke	[80–82]

**Table 3:** Summary of outcomes of Tai Chi interventions in stroke recovery.

Intervention methods	Course of disease	Number of cases	Randomized trial	Comparator	Intervention time	Positive findings
Chen styles of Tai Chi	0.25–12 months	40	Yes	Modern rehabilitation therapy	20–40 minutes/time, 5 times/week, 0.5 month	Chen styles of Tai Chi-style Tai Chi, fixed-foot stance Yunshou, modified Tai Chi, and Tai Chi. It can significantly improve patients' motor function, balance and coordination ability, cognitive function, nerve excitability, daily living ability, emotional regulation, and cardiopulmonary function and has a certain safety and prevention of falls. With the prolongation of intervention time, the effect is more obvious. The curative effect of Tai Chi combined with modern rehabilitation technology is better than that of modern rehabilitation technology alone, and the curative effect is improved with the prolongation of intervention time. Tai Chi has certain safety and prevents falls
Fixed-foot stance Yunshou	<6 months	60	Yes	Routine treatment and rehabilitation nursing	30 minutes/time, 5 times/week, 2 months	
Fixed-foot stance Yunshou combined with bobath handshake training	<6 months	59	Yes	Routine treatment and rehabilitation nursing	30 minutes/time, 5 times/week, 2 months	
Tai Chi Yunshou	<6 months	60	Yes	Routine treatment and rehabilitation nursing	30 minutes/time, 1 time/week, 5 days/week, 2 months	
Tai Chi Yunshou	>3 months	30	Yes	Basic therapy (conventional internal medicine and health education)	60 minutes/time, 1 time/day, 5 days/week, 3 months	
Modified Tai Chi	0.5–2 months	62	Yes	Stretching training	30 minutes/time, 1 time/day, 5 days/week, 1 month	
Modified Tai Chi	<6 months	73	Yes	Modern rehabilitation therapy	60 minutes/time, 1 time/day, 5 days/week, 1 month	
Modified Tai Chi	<6 months	22	Yes	Routine rehabilitation	60 minutes/time, 1 time/day, 5 days/week, 1 month	
Modified Tai Chi	<6 months	40	Yes	Routine rehabilitation	60 minutes/time,1 time/day,5 days/week,1 month	
Tai Chi Yunshou	>3 months	80	Yes	Routine rehabilitation	60 minutes/time, 1 time/day, 5 days/week, 3 months	
Tai Chi	≥3 months	17	Yes	Traditional rehabilitation	60 minutes/time, 1 time/day, 2 days/week, 6 months	
Tai Chi catwalk exercise combined with acupoint tuina	0.5–6 months	180	Yes	Traditional Chinese and western medicine in combination with comprehensive rehabilitation	30 minutes/time, 2 times/day, 6 months	
Taijiquan	>3 months	62	Yes	Modern comprehensive rehabilitation treatment	40 minutes/time, group training 3 times/week, individual training 2 times/week, 2 months	
Taijiquan	≥3 months	16	Yes	Traditional rehabilitation	60 minutes/time, group training 1 time/week, training in family 1 time/week, 6 months	
Taijiquan	>0.5 month	56	Yes	Routine rehabilitation	30 minutes/time, 1 time/day, 5 days/week, 1 month	
Tai Chi posture training	<6 months	110	Yes	Modern rehabilitation therapy	60 minutes/time, 1 time/day, 5 days/week, 1 month	
Tai Chi pile work	0.5–3 months	80	Yes	Physical therapy and homework therapy	20 minutes/time, 2 times/day, 3 months	
Modified 24 styles of Tai Chi	<6 months	60	Yes	Antidepressant drug treatment	60 minutes/time, 1 time/day, group training 1 day/week, 3 months	
Modified 24 styles of Tai Chi	<3 months	105	Not clear	Control or Baduanjin	40 minutes/time, group training 3 times/week, individual training 2 times/week, 2 months	
Body weight support (BWS)and Tai Chi	≥3 months	71	Yes	Conventional rehabilitation therapies	40 minutes/time, 3 times/week, 3 months, 20 minutes/BWS, 20 minutes/Taichi	
Community-basedYang-style Tai Chi	≥3 months	28	Yes	Usual care	60 minutes/time, 3 times/week,3 months, a 20 minutes warm-up period, 30 minutes of Tai Chi exercise, and a 10 minutes cool-down period	
Yang-style24-postureshort-form Tai Chi	≥3 months	145	Yes	SilverSneakers, usual care	60 minutes/time, 3 times/week, 3 months, a 10 minutes warm-up period, 40 minutes of Taichi exercise, and a 10 minutes cool-down period	
Tai Chi Yunshou exercise	≥3 months	244	Yes	Rehabilitation	60 minutes/time, 5 times/week, each session comprised 45 minutes of exercise plus a 15 minutes warm-up and cool down. 3 months	
Tai Chi	≥3 months	16	Yes	Traditional rehabilitation	6 months	

*Note.* The column of course of disease is based on month, and those less than 1 month are converted proportionally; in the column of intervention time, the time of each intervention is calculated as minutes, and the total time of intervention is calculated as months. Each exercise therapy status analysis in TCMET was expressed in such a discounted way in terms of the course of disease and intervention time.

**Table 4:** Summary of outcomes of Baduanjin interventions in stroke recovery.

Intervention methods	Course of disease	Number of cases	Randomized trial	Comparator	Intervention time	Positive findings
Baduanjin combined with Traditional Chinese medicine measures	<6 months	90	Yes	Traditional Chinese medicine measures	30 minutes/time, 1 time/day, 6 months	The combination of Baduanjin, eighteen section brocade, and other methods can effectively improve the overall clinical efficacy of stroke recovery patients; improve neurological function and limb function; reduce the degree of depression of patients; improve motor function, muscle strength, muscle tone, life independence ability, and balance ability; and improve overall cognitive function, cognitive dysfunction execution, attention, memory, and processing speed
Baduanjin combined with action observation therapy	<3 months	90	Yes	Routine treatment and nursing plan/Baduanjin	20 minutes/time, 1 time/day, 6 days/week, 1 month	
Baduanjin combined with balancing function training	<6 months	60	Yes	Balancing function training	20 minutes/time, 2 times/day, 1.5 months	
Baduanjin combined with balancing training	1–3 months	62	Yes	Balance training	20 minutes/time, 2 times/day, 5 days/6 days, 1.6 months	
Baduanjin combined with rehabilitation training	<6 months	224	Yes	Rehabilitation training	20 minutes/time, 2 times/day, 7 days/week, 1.5 months	
Baduanjin exercise	≥2 months	48	Yes	Health education	40 minutes/time, 3 times/week, 6 months	
Baduanjin exercise	≥2 months	48	Yes	Health education	40 minutes/time, 3 times/week, 6 months	
Baduanjin	1–6 months	60	Yes	Control group	45 minutes/time, 3 times/week, a 5 minutes warm-up period, 5 minutes relaxation period two times, 1 month	
JieYu no. 1 recipe combined with Baduanjin	<3 months	80	Yes	Sertraline hydrochloride	20 minutes/time, 2 times/day, 5 days/week, 1 month	
Eighteen-section brocade combined with routine care and rehabilitation	0.5–6 months	80	Yes	Routine care and rehabilitation	30 minutes/time, 2 time/day, a 5 minutes warm-up period, 2 months	
Eighteen-section brocade combined with rehabilitation	0.25–6.25 months	96	Yes	Rehabilitation	30 minutes/time, 2 time/day, 3 months	
Cluster needling technique at the head point and Baduanjin exercise	1–3 months	60	Yes	Cluster needling technique at the head points	20 minutes/time, 2 times/day, 5 days/week, 1.5 months	
Five-element music therapy combined with Baduanjin	6.35 ± 1.69^*∗*^ months	72	Yes	Baduanjin	30 minutes/time, 2 time/day, 1.3 months	
Acupuncture combined with eighteen-section brocade	<3 months	201	Yes	Routine therapy	30 minutes/time, 2 time/day, 1 months	
Zishen Yisui acupuncture based on the Baduanjin	3–12 months	80	Yes	Baduanjin exercise	40 minutes/time, 3 times/week, 2 months	
Baduanjin exercise	6.58 ± 2.14^*∗*^ months	48	Yes	Health education sessions	40 minutes/day, 3 days/week, 6 months	
Baduanjin Qigong	>3 months	58	Yes	2 sessions of supervised conventional fitness training in the first week combined with home-based exercise practice	50 minutes/time, 3 times/week, a 10 minutes warm-up, 10 minutes cool down, 4 months	
Baduanjin exercise based on original medication and rehabilitation treatment	>3 months	48	Yes	Original medication and rehabilitation treatment	40 minutes/day, 3 days/week, 6 months	

*Note.* ^*∗*^indicates that the course of the disease was found in baseline data and expressed as a mean, not clearly defined in the inclusion criteria.

**Table 5:** Summary of outcomes of Daoyin interventions in stroke recovery.

Intervention methods	Course of disease	Number of cases	Randomized trial	Comparator	Intervention time	Positive findings
Daoyin method of general treatise on causes and manifestations of all diseases	≤6 months	68	Yes	Routine rehabilitation	40 minutes/day, 5 days/week, 1.5 months	Daoyin can improve upper limb motor function, balance and coordination, daily living ability, and neurological function in stroke patients
Daoyin method of general treatise on causes and manifestations of all diseases	<6 months	60	Yes	Routine rehabilitation	30 minutes/time, 2 times/day, 5 days/week, 1.5 months	
Daoyin method of Chao Yuanfang	<12 months	130	Yes	Routine rehabilitation	5 days/week, 0.75 month	
Daoyin method of Chao Yuanfang	<6 months	40	Yes	Routine rehabilitation	20 minutes/time, 2 times/day, 6 days/week, 0.5 month	
Daoyin method of Chao Yuanfang combined with routine rehabilitation	<6 months	40	Yes	Routine rehabilitation	20 minutes/time, 2 times/day, 6 days/week, 0.5 month	
Daoyin method of Chao Yuanfang	<6 months	30	Yes	Routine rehabilitation	20 minutes/time, 2 times/day, 6 days/week, 0.5 month	
Daoyin therapy and routine rehabilitation training	1–6 months	60	Yes	Routine rehabilitation training	45–60 minutes/time, 1 time/day, 5 days/week, 1.5 months	
Daoyin therapy and routine rehabilitation training	0.5–2 months	200	Yes	Routine rehabilitation	45–60 minutes/time, 1 time/day, 1.5 months	
Upper limb guiding technique	4.29 ± 1.87^*∗*^ months	90	Yes	Bobath therapy	30–45 minutes/time, 1.5 months	

*Note.* ^*∗*^indicates the same comments as Table 4.

**Table 6:** Summary of outcomes of six-character tip interventions in stroke recovery.

Intervention methods	Course of disease	Number of cases	Randomized trial	Comparator	Intervention time	Positive findings
Six-character tips	>0.5 months	34	Yes	Routine treatment, nursing, and rehabilitation	18–24 minutes/time, 1 time/day, 7 days/week, 3 months	Six-character tips combined with routine rehabilitation, basic pronunciation training, and traditional breathing exercise can significantly improve pulmonary respiratory function, speech disorders, daily living ability, motor function, balance and coordination, cognitive function, nerve damage, depression, etc.
Six-character tips combined with conventional articulation training	0.5–6 months	157	Yes	Traditional breathing training and conventional articulation training	20 minutes/time, 1 time/day, 5 days/week, 0.5 month	
Six-character tips	<6 months	60	Yes	Routine care for depression after stroke	15–20 minutes/time, 2 times/day, 0.93 month	
Liu Zi Jue qigong with basic articulation training	0.5–6 months	60	Yes	Traditional breathing training + basic articulation training	20 minutes/time, 5 times/week, 0.75 month	
Six-character tips	≤3 months	84	Yes	Routine treatment and care	30 minutes/time, 1 time/day, 5 days/week, 3 months	
Six-character tips combined with the diaphragm muscle release technique	3–7 months	80	No	Routine rehabilitation such as inhalation training	30 minutes/time, 1 time/day, 5 days/week, 2 months	
Liu Zi Jue qigong combined with conventional rehabilitation training	0.5–6 months	160	Yes	Traditional core stability training combined with routine rehabilitation	15 minutes/time, 1 time/day, 5 days/week, 0.5 month	
Six-character tips combined with inspiratory muscle training	3.61 ± 2.35^*∗*^ months	75	Yes	Routine rehabilitation/routine inspiratory muscle training	30 minutes/time, 1 time/day, 5 days/week, 3 months	
Liu Zi Jue qigong combined with conventional breathing speech training	4–14 months	50	Yes	Conventional breathing speech training	20 minutes/time, 1 time/day, 5 days/week, 1 month	
Six-character formula respiratory gymnastics	1–12 months	68	Yes	Medical treatment, routine rehabilitation, and occupational therapy	30 minutes/time, 1 time/day, 5 days/week, 3 months	

*Note.* ^*∗*^indicates the same comments as Table 4.

**Table 7:** Summary of outcomes of Yi Jin Jing, five-fowl play, and relaxation exercise interventions in stroke recovery.

Intervention methods	Randomized trial	Comparator	Intervention time	Positive findings
Yi Jin Jing(Yi Jin Jing, modified Yi Jin Jing, Yi Jin Jing + Xingnao kaiqiao acupuncture, Yi Jin Jing + acupuncture)	Yes	Routine rehabilitation/group occupational therapy/basic treatment/acupuncture	20–60 minutes/time, 1 time/day, 3–6 times/week, 0.7–3 months	Yi Jin Jing combined with acupuncture and routine rehabilitation can significantly improve motor function, daily living ability, cognitive function and emotional state of stroke patients
Five-fowl play	Yes	Routine rehabilitation	30–60 minutes/time, 5 times/week, 1–5 months	It can significantly improve the motor function, daily living ability, and balance and coordination of patients with stroke hemiplegia
Relaxation exercises (relaxation exercises + rehabilitation and relaxation exercises + bobath therapy)	Yes	Routine rehabilitation/rehabilitation care and health education/bobath therapy + basic rehabilitation	20–30 minutes/time, 1 time/day, 1–2 months	Relaxation exercise combined with routine rehabilitation can improve motor function, neurological function impairment, depression and daily living ability of stroke patients with hemiplegia during recovery, and the effect is better than that of conventional rehabilitation alone

## Data Availability

All data supporting the findings of this study are available within the article.
